This article has been retracted.

# Reduced expression of Jak-1 and Tyk-2 proteins leads to interferon resistance in Hepatitis C virus replicon

**DOI:** 10.1186/1743-422X-4-89

**Published:** 2007-09-18

**Authors:** Sidhartha Hazari, Lizeth Taylor, Salima Haque, Robert F Garry, Sander Florman, Ronald Luftig, Frederic Regenstein, Srikanta Dash

**Affiliations:** 1 Department of Pathology and Laboratory Medicine, Tulane University Health Sciences Center, 1430 Tulane Avenue, New Orleans, USA; 2 Microbiology and Immunology, Tulane University Health Sciences Center, 1430 Tulane Avenue, New Orleans, USA; 3 Medicine, Tulane University Health Sciences Center, 1430 Tulane Avenue, New Orleans, USA; 4 Surgery, Tulane University Health Sciences Center, 1430 Tulane Avenue, New Orleans, USA; 5 Department of Microbiology, Immunology and Parasitology, Louisiana State University Health Sciences Center, New Orleans-70112, USA; 6 Louisiana State University-International Center of Medical Research and Training, University of Costa Rica, Costa Rica

## Abstract

**Background:**

Alpha interferon in combination with ribavirin is the standard therapy for hepatitis C virus infection. Unfortunately, a significant number of patients fail to eradicate their infection with this regimen. The mechanisms of IFN-resistance are unclear. The aim of this study was to determine the contribution of host cell factors to the mechanisms of interferon resistance using replicon cell lines.

**Results:**

HCV replicons with high and low activation of the IFN-promoter were cultured for a prolonged period of time in the presence of interferon-alpha (IFN-alpha2b). Stable replicon cell lines with resistant phenotype were isolated and characterized by their ability to continue viral replication in the presence of IFN-alpha. Interferon resistant cell colonies developed only in replicons having lower activation of the IFN promoter and no resistant colonies arose from replicons that exhibit higher activation of the IFN promoter. Individual cell clones were isolated and nine IFN resistant cell lines were established. HCV RNA and protein levels in these cells were not altered by IFN- alpha2b. Reduced signaling and IFN-resistant phenotype was found in all Huh-7 cell lines even after eliminating HCV, suggesting that cellular factors are involved. Resistant phenotype in the replicons is not due to lack of interferon receptor expression. All the cell lines show defect in the JAK-STAT signaling and phosphorylation of STAT 1 and STAT 2 proteins were strongly inhibited due to reduced expression of Tyk2 and Jak-1 protein.

**Conclusion:**

This in vitro study provides evidence that altered expression of the Jak-Stat signaling proteins can cause IFN resistance using HCV replicon cell clones.

## Background

Hepatitis C virus (HCV) is a blood-borne human pathogen. There are 170 million people worldwide infected with HCV, representing a significant public health problem. Only a small fraction of individuals develop immunity and clear virus infection naturally. The majority of people exposed to HCV slowly develop into chronic infection. Long-standing chronic inflammation in the liver due to the virus infection leads to liver cirrhosis and carcinoma [1-7]. Infection with HCV is the leading cause of liver transplantation in the United States [8]. Standard therapy for chronic HCV infection is a combination of IFN-α and ribavirin, but the majority of chronic hepatitis C patients cannot clear their infection with this regimen. Patients infected with genotype 1 HCV in the United States are frequently resistant to IFN-α and ribavirin treatment [9-13]. The reason why some chronic hepatitis C patients do not respond to interferon therapy is unknown.

The HCV belongs to the family *Flaviviridae*. There are six different genotypes of HCV distributed worldwide with more than 50 subtypes [14,15]. There is 30% sequences variation among each genotype, 15% among sub-types and 1–5% among quasisspecies. The organization of HCV RNA genome among all genotypes is similar. It begins with a 5'untranslated region (UTR), long-open reading frame and a 3' UTR region [16]. The HCV genome encodes a large polyprotein of 3000 amino acids, which is processed into structural and non-structural protein in the infected cells by viral and cellular proteases. Some reports demonstrate that certain genotypes of HCV respond better to interferon therapy compared than others. For an example, 80% of chronic hepatitis C patients infected with genotype 2 and 3 can clear the virus infection, while only 50% in patients infected with genotype 1 [17,18] show a sustained virological response. This clinical observation suggests the involvement of viral factors in response to interferon therapy. A number of molecular studies have been performed with results suggesting that some of the HCV structural and/or non-structural viral proteins block the interferon induced antiviral pathways [19-26]. The molecular basis of HCV resistance to interferon has focused on NS5A and E2 protein action on the interferon induced protein kinase R [27-31]. Recent studies also suggest that the HCV protease (NS3/NS4A) can block the production of endogenous of IFN-beta [32]. Most of the studies of IFN resistance have focused on virus-related factors, and little attention has been paid to host factors. The underlying mechanisms of interferon resistance against chronic hepatitis C are not yet clear. The HCV RNA replicon systems have now proved to be a suitable model to study the host-virus interaction. Understanding how viral and host factors influence interferon sensitivity is important as it may lead to the development of alternative strategies to improve the success rate of interferon based antiviral therapy.

Interferons are a family of cytokines that play a very important role in innate immunity and protect humans from infections with number of viruses and intracellular organisms [33]. The interferon system is activated during viral infection of a host cell, thus inhibiting virus replication during the host innate immune response. There are two types of interferon. Type I interferon includes IFN-α and interferon beta (IFN-β) and Type II interferon includes interferon gamma (IFN-γ). Since endogenous interferon produced by the infected cell is not sufficient to eliminate the infection, exogenous recombinant human IFN-α has been therefore used to treat chronic hepatitis C. The cloning and sequencing of functional cDNAs for each interferon has made it possible to use this cytokine as a potential antiviral to treat number of virus infections [34]. The antiviral action of interferon is initiated when IFN-α binds the receptor. Interferon binding to the cell surface receptors activates the intracellular signaling pathways, which involve Janus kinase (JAK1), tyrosine kinase 2 (TYK2) and signal transducer and activator of transcription (STAT1 and STAT2) proteins. The JAKs phosphorylate STAT proteins that either homo-or heterodimerize and translocate to the nucleus thus inducing the expression of the IFN-stimulated genes (ISG). The phosphorylated STAT1 and STAT2 combine with IRF-9 (interferon regulatory factor 9) to form a trimeric ISGF-3 complex. This complex enters the nucleus and binds to a consensus DNA sequence [GAAAN(N)GAAA] called the interferon stimulated response element (ISRE) [35,36]. This regulatory sequence is present upstream of most IFN-α and IFN-β responsive genes. These cascades of molecular signaling are essential for stimulation of interferon mediated gene transcription. Previous studies in our laboratory suggest that activation of interferon stimulated responsive element (IFN-promoter) is critical in a successful antiviral response against hepatitis C. This activation of interferon induced gene activation via JAK-STAT pathways varies among different Huh-7 clones [37].

This study was initiated to define the significance of IFN-promoter activation in different replicon cell lines with respect to the antiviral action of IFN-α2b. We found that replicon cell lines with a low-level induction of interferon promoter frequently develop resistance to IFN-α. In this report, we have developed several stable replicon cell lines in which replication of HCV is totally resistant to IFN-α. The role of viral and cellular factors in the mechanisms of IFN-resistance was examined. We showed here that the altered expression of proteins in the Jak-Stat signaling pathway of replicon cells block IFN-induced gene activation and cause interferon resistance.

## Results

### Isolation of interferon resistant HCV replicon cell lines

Previously, we reported data suggesting that activation of this ISRE-promoter is important for a successful antiviral action of IFN-α in replicon cells (37). It was observed that the level of expression of luciferase from IRES promoter by interferon varies among HCV replicon cell clones. To understand the significance of this observation, we performed the present study to determine whether the differences in the level of ISRE-promoter (IFN-promoter) activation among different replicon cells are related to interferon sensitivity. Three different replicon cell lines showing lower ISRE promoter activation (Con-15, Con-17 and Con-24) and three replicon cell line with higher ISRE promoter activation (5–15, 9–13 and KR) were treated with IFN-α2b (10–1000 IU/ml) and cultured in the medium containing G-418 (1 mg/ml). All six replicon cell lines used in our experiments have been prepared using prototype Con1 sub-genomic replicon HCV RNA (Fig. 1A). The HCV replicon is a dicistronic chimeric RNA which contains the gene encoding for neomycin phosphotransferase (conferring resistance to G-418) downstream of the HCV IRES. The second cistron in the same RNA contains encephalomyocarditis virus IRES sequences for efficient translation of HCV non-structural proteins and this chimeric RNA terminates with the HCV 3'UTR. This sub-genomic RNA replicates at a high level in Huh-7 cells and cell colonies develop that are resistant to G-418. The ability of HCV sub-genomic RNA to replicate and form G-418 cell colonies in the presence and absence of IFN-α was examined. IFN-α efficiently inhibited HCV RNA replication in three replicon cell lines with higher activation of ISRE promoter and there were no viable cell colonies are formed. However, antiviral action of interferon against HCV was partially effective in the cell line having lower activation of ISRE promoter since many visible clones were found (Fig. 2). The cell clones that survived interferon treatment grew well in the presence of interferon alpha. Individual clones were picked and nine different stable cell lines from each low inducer replicon [Con-15 (15/1, 15/2, 15/3), Con-17 (17/1, 17/2, 17/3) and Con-24 (24/1, 24/2, 24/3)] were prepared. The nine different replicon cell lines were maintained in the presence of IFN-α2b (1000 IU/ml) for prolonged periods to make sure that they are truly resistant to interferon.

**Figure 1:** **Diagram of the sub-genomic replicon and reporter plasmid constructs used in the experiments**. (A) The HCV replicon is a dicistronic chimeric RNA which contains the gene encoding for neomycin phosphotransferase downstream of the HCV IRES. The second cistern in the same RNA contains EMCV-IRES sequences for efficient translation of HCV non-structural proteins and this chimeric RNA terminates with the HCV 3'UTR. This sub-genomic clone has adaptive mutation S1179I that allows high level replication of RNA in Huh-7 cells and cell colonies develop that are resistant to neomycin. (B) pISRE-Luc reporter plasmid construct containing firefly luciferase reporter gene used to measure IFN-promoter activation in replicon cell lines. This construct has four copies of ISRE sequences positioned up stream of Herpes simplex virus thymidine kinase promoter TATA box, which drives the expression of firefly luciferase. (C) Represents monocistronic reporter constructs that express green fluorescent protein translated by HCV IRES by using a T7 inducible system.

**Figure 2:** **Isolation of HCV replicon cell lines possessing IFN-resistant phenotype**. Three stable replicon cell lines (Con-24, Con-17 and Con-15) having low ISRE-promoter activation and three replicon cell lines (9/13, 5/15 and KR) with high ISRE promoter activation were treated with or without interferon alpha 2b (1000 IU/ml) for 4 weeks in a growth medium containing G-418 (1 mg/ml). The ability of replicon cells to develop G-418 resistant cell colonies was examined. Cell colonies were developed only in low ISRE replicons. Three individual colonies from each dish were picked up and nine stable cell lines were generated.

### Characterization of HCV replicon cell lines

The antiviral effect of IFN-α against HCV in nine resistant-replicon cell line was confirmed by measuring their ability to form cell colonies in a medium containing G-418, sustained viral RNA replication and protein expression. All nine replicon cell lines were cultured in a medium containing 1 mg/ml of G-418 in the presence of cyclosporine-A or IFN-α. Their ability to form G-418 cell colonies was measured in 100-mm tissue culture dishes. Results shown in Fig. 3A, indicate that all resistant replicon cell lines grew in the presence of IFN-α but not in the presence of Cyclosporine-A. It is known that Cyclosporine-A inhibit HCV RNA replication in Huh-7 cells by a different mechanism independent of Jak-Stat pathway. There is one report documenting that replication efficiency depends upon cell proliferation. To examine the possibility that interferon resistance phenotype seen in the replicon cells is due to certain growth advantage as compared to sensitive cells, growth rate of nine different replicon cells were over one week was compared to sensitive cell lines. No significant differences in cell growth were observed between nine different resistant cell lines and five different sensitive cell lines.

**Figure 3:** **Three panels showing HCV replication and protein expression in IFN resistant replicon cell lines**. (A) Shows growth of nine different HCV replicon cell lines in medium containing 1 mg/ml G-418 in the presence of IFN-α2b. All cell lines grew and formed IFN-resistant cell colonies. Cyclosporin-A (1 mg/ml) inhibited the colony formation in the replicon cell lines in presence of G-418. (B) HCV replication is resistant to IFN-α2b treatment in nine different replicon cell lines. Stable cell lines were treated with or without IFN-α2b (1000 IU/ml) and cyclosporine-A (1 mg/ml) for a week. Intracellular HCV positive strand RNA was measured by RPA using an antisense riboprobe targeted to the 5'UTR. (C) Shows the effect of IFN-α2b on NS3 protein expression in interferon sensitive versus interferon resistant cell clones. Replicon cells in chamber slides were treated with IFN-α2b (1000 IU/ml) for a week, and immunostaining for NS3 protein was performed using a monoclonal antibody. IFN treatment abolished NS3 protein expression in sensitive cells (S-5/15). No inhibition was seen in any of these three resistant cell lines (R-Con-15, R-Con-17 and R-Con-24).

To make sure that intracellular HCV RNA levels are steadily maintained in the interferon treated cells, total RNA was isolated from each replicon cell line and subjected to RPA assay using probe targeted to the 5' UTR. Results of this experiment (Fig 3B) indicated that the 296 nucleotides protected band was detectable in all resistant cell lines. There were no differences in the HCV RNA levels between cells that were treated with or without interferon. Intracellular HCV RNA levels in the nine different replicon cells were examined by RPA assay after Cyclosporine-A treatment. The level of HCV protein expression was compared between sensitive and resistant replicon cells after interferon treatment by immunocytochemical staining using a monoclonal antibody to NS3 protein. Results of this experiment are shown in (Fig. 3C) indicating all resistant cells maintain high levels of viral protein expression after interferon treatment.

### Interferon resistant replicons showed reduced IFN-signaling

We reasoned there might be two possibilities that could contribute to the IFN-resistant phenotypes in the cell culture models. First possibility is that sustained expression of viral proteins directly block Jak-Stat signaling and make cells insensitive to interferon. The second possibility is that there may be a defect at the level of intracellular signaling of interferon in these replicons. We have showed earlier that IFN-α successfully inhibits translation and replication of full-length as well as sub-genomic HCV RNA in Huh-7 cells suggesting that viral protein expression did not inhibit interferon action. To clarify the role of cellular contribution in the mechanism of IFN-resistance, HCV replication was eliminated from each cell line by treatment with Cyclosporine-A. The success of Cyclosporine-A treatment and absence of HCV RNA in these cured cells was confirmed by RPA and immunostaining for HCV NS3 protein. Cured cell lines were prepared from each resistant replicon and cultured in regular growth medium without G-418. Interferon signaling pathway in cured replicon cells was examined using a construct pISRE-luciferase reporter plasmid (Fig. 1B) in a transient transfection assay. Results obtained from those experiments suggested that luciferase activity in all the nine different replicon cells were significantly low as compared to the interferon sensitive cell lines (Fig. 4). The differences in the results of luciferase expression from the ISRE promoter between IFN-sensitive and IFN-resistant cells are found to be statistically significant (p < 0.05).

**Figure 4:** **IFN signaling in established replicon cell lines**. Each cured IFN resistant and sensitive cell lines were transfected with the pISRE-Luc plasmid. The activation of IFN promoter in the replicon cell lines was determined in the presence or absence of IFN-α2b (1000 IU/ml) after 24 hours. All nine interferon resistant cell lines have lower activation of IFN-promoter as compared to interferon sensitive cell lines.

We reported previously that interferon inhibits HCV replication by blocking at the level of viral IRES mediated translation using a green fluorescence protein based sub-genomic expression system [37,38]. Experiments were performed to determine whether green fluorescence expression from HCV IRES sub-genomic clone inhibited by IFN-α in these cells. Nine different cured IFN-resistant Huh-7 cell lines were transfected with HCV IRES-GFP plasmid using a two-step transfection procedure described in our previous publications. The cells were cultured in the presence and absence of IFN-α (1000 IU/ml). The expression of green fluorescence between IFN-resistant and sensitive cells was examined under a fluorescence microscope. Results of these experiments indicate that HCV IRES mediated translation is not sensitive to IFN-α in all resistant Huh-7 cells (Fig. 5). Interferon effectively inhibited expression of HCV IRES-GFP in all IFN-sensitive clones. These results led us to conclude that these nine different cell lines that show interferon resistant phenotypes have defects in the interferon signaling.

**Figure 5:** **Interferon action on the IRES-mediated translational inhibition was prevented in cured resistant cell lines**. Effect of interferon on IRES-GFP translation regulation was examined using one cured sensitive and nine resistant Huh-7 cell lines. Cells were transfected with IRES-GFP plasmid and treated with 1000 IU/ml interferon alpha. After 24 hours, GFP expression was recorded. Cured cells prepared from resistant clones unable to activate interferon signaling and no inhibition of HCV IRES was seen.

### Defective Jak-Stat signaling in resistant replicons

We performed experiments to compare the level of expression of individual proteins of Jak-Stat pathways between IFN-sensitive and IFN-resistant cells. Interferon first binds to cell surface receptor that leads to activation of down stream Jak-Stat signaling and activation of antiviral genes. First we determined whether the interferon resistant phenotypes in these cells is due lack of expression of functional interferon receptors on the cell surface. To test this possibility, we performed a binding assay using ^125^I-labeled interferon and nine different cured resistant cell lines. The binding assay results were compared with a cured interferon sensitive cell line to see the differences (Fig. 6). It was observed that all resistant and sensitive Huh-7 cells equally bind to ^125^I- IFN-α. The amounts of ^125^I-IFN bound (cpm) to the resistant cell line (15-1, 15-2 and 15-3) are comparable to sensitive cells (Fig. 6A). Similar results were obtained with 17-1, 17-2 and 17-3 (Fig. 6B) and 24-1, 24-2, 24-3 (Fig 6C). The receptor binding studies were also confirmed by examining expression of interferon receptors using protein lysates by western blot analysis (Fig. 7). Results of these experiments suggest that the defect in the interferon signaling is not due to a lack of cell surface expression of receptors.

**Figure 6:** **IFN receptor binding affinity between sensitive and resistant Huh-7 cell lines**. Equal numbers of cured cells were incubated with different concentrations (3.9 to 125 ng) of ^125^I-IFN-α2b at 37°C for one hour. Non-specific binding was measured in presence of 100-fold excess of unlabeled IFN-α2b for each dilution. Cells were washed twice in PBS. Radioactivity (cpm) of each cell pellet was measured. The amount of interferon specifically bound was determined by subtracting non-specific binding from total binding. Specific binding of ^125^I-IFN-α2b to three groups of resistant cell lines and one sensitive cell line are shown (A-D).

**Figure 7:** **Western blot analysis of the Jak-Stat signaling pathway in IFN-sensitive and IFN-resistant cell lines**. Three representative cured Huh-7 clones of IFN-resistant and one Huh-7 clone of IFN-sensitive cell line were treated with IFN-alpha (1000 IU/ml) for 30 minutes. Cell lysates were prepared and then equal amounts of protein lysates were used to examine the expression of IFN-receptor (IFNAR1), Jak-1, Tyk2, Stat 1, Stat 3 and Stat 3, phosphorylated Stat 1 and Stat 2 by Western blot analysis. Beta actin levels were used, as a control to make sure that equal amount of protein was present in the extracts. All IFN-resistant cell lines have reduced expression of Tyk2 and showed lack of Stat phosphorylation.

We then examined whether there is an alteration in the expression of down-stream signaling proteins that could explain the cause of reduced IFN-signaling. Protein lysate was made from three IFN-resistant cell lines (R-Con-15/1, R-Con-17/1 and R-Con-24/1) (representative of each series) and one sensitive replicon cell line. Equal amounts of protein extracts were examined for the expression of Jak-1, Tyk-2, Stat1, Stat 2 and Stat3 by Western blot analysis. The expression of unphosphorylated IFNAR1, Jak-1, Tyk2, Stat1, Stat2 and Stat3 protein between IFN-sensitive and IFN-resistant cells is shown in Fig. 7A. The results of this experiment revealed that all resistant replicon cell lines we developed have reduced expression of Tyk2 as compared to the sensitive replicon cells. In some resistant replicons expression of Jak-1 was also reduced. There were no differences in the expression of Stat 1 and Stat 2 proteins between sensitive and resistant cells.

Interferon treatment leads to tyrosine phosphorylation of Stat 1 and Stat 2 protein followed by heterodimerization of Stat1 and Stat 1. This dimer then enters the nucleus to drive the transcription of antiviral genes. Therefore, phosporylation status of Stat1 and Stat 2 proteins between IFN-sensitive and resistant replicon cells was examined using phosphorylation specific commercially available antibodies (Fig. 7B). It was observed that phosphorylation of Stat1 and Stat2 was strongly inhibited in all interferon resistant replicons as compared to the IFN-sensitive replicon. The differences seen in our analysis is not due to the differences in the amount of proteins loaded into the gel since beta-actin levels are found to be similar.

## Discussion

Interferon alpha in combination with ribavirin is the standard treatment for patients with chronic hepatitis C virus infection. This therapy can eliminate virus infection in approximately 80% of patients infected with genotype 2 or 3, and 50% in patients infected with genotype 1. The reason why many patients infected with genotype 1 virus fail to eradicate the virus is not clear. The mechanisms of the resistance may be multifactorial. Several molecular studies have been performed indicating that the viral factor plays a role in the persistent hepatitis C virus infection and interferon resistance. Results of these studies indicate that full-length as well as individual proteins of HCV (NS5A, Core, NS3 and E2) block interferon action. Among all the viral proteins studied the NS5A protein of HCV has been proposed to be crucial for determining interferon sensitivity. Chronic hepatitis C patients showing amino acid substitution in the IFN-sensitivity determining region (2209–2248) of NS5A was found to have a good response to interferon therapy. The role of ISDR mutation and mechanisms of interferon resistance is not yet conclusive. In contrast, clinical observations have suggested that host factors may also play roles in IFN response [39,40].

In this report, we used hepatic cell lines replicating sub-genomic RNA since they represent similar to chronically infected liver cells. Different laboratories including our own have used the replicon based cell lines to test interferon action against HCV replication. Results of all these studies now suggest that interferon can successfully inhibit replication of HCV sub-genomic RNA. Interferon treatment activates a cascade of signal transduction pathways through its cell surface receptors that stimulate synthesis of numerous antiviral genes. This signaling cascade involves cell surface receptors, Janus kinase (Jak-1) and tyrosine kinase 2 (Tyk-2) and signal transducer and activator of transcription (STAT1 and STAT2) proteins. The Jak-1 and Tyk-2 phosphorylate the STAT proteins which either homo-or heterodimerizes and then translocates to the nucleus and then binds to a consensus DNA sequence called the interferon stimulated response element (ISRE). This regulatory sequence is present upstream of most IFN-α and IFN-β responsive genes. These cascades of molecular signaling are essential for the stimulation of interferon mediated gene transcription. To support this notion we previously showed that interferon alpha treatment activates the ISRE promoter driven transcription of luciferase gene by transient transfection experiments and the pathways that leading to IFN-promoter activation also varies among different replicon cell lines [37].

To understand the significance of IFN-promoter activation and interferon resistance in replicon cell lines, we treated high and low inducer replicon cell lines with IFN-α2b for a prolonged period of time with varied amount of IFN starting from 10 IU to 1000 IU/ml. It was found that cells that show a low level of IFN-promoter activation could not eliminate HCV replication in all cells since some Huh-7 clones develop resistance to interferon. Using this approach, we developed interferon resistant cell lines by treating low inducer replicon cells with alpha interferons. We showed clearly that all these resistant replicons have sustained viral replication that cannot be inhibited by alpha interferon. The intracellular HCV RNA levels and protein levels did not alter after interferon treatment. We clarified that viral factors do not contribute to the acquisition of IFN-resistance in these replicon cells since the cured cells prepared from each replicon still show reduced IFN signaling. Interferon signaling in the cured cells was determined using a luciferase based reporter assay. It was determined that there were no differences in the level of IFN-promoter activation in all resistant cell lines with or without HCV replication. Based on these evidences the role of virus contribution to the mechanisms of IFN-resistance in replicons was excluded. Expression of GFP from HCV IRES was examined between sensitive and resistant in the presence of interferon and found that HCV IRES translation is not inhibited in resistant Huh-7 cells. These results indicated that interferon resistant phenotypes associated in our replicon cell line might be due to a specific defect in the IFN-signaling pathways.

To identify the defect that is responsible for reduced interferon signaling in these replicon cells, expression of Jak-Stat proteins of interferon was examined. Interferon signaling occurs through a series of protein-protein interactions that initiate through a cell surface receptor expression. We examined the expression of interferon receptor expression by Western blot analysis as well as by using receptor-binding assay. All the nine resistant cell lines bind to iodinated IFN-α. It was determined that the nature of the defect is not due to the lack of expression of functional receptors on the cell surface. We then examined the expression of the down-stream signaling protein of the Jak-Stat pathway between IFN-sensitive and resistant replicons. An equal amount of protein lysates were first tested for beta actin levels to exclude the possibility that differences are not due to a lack of adequate amounts of protein in the extracts. It was found that all resistant Huh-7 cells have reduced expression of Tyk2. Reduced expression of Jak-1 was also observed in some resistant Huh-7 cells. The levels of Stat1 and Stat2 expression was found be similar between resistant and sensitive replicons. The phosphorylation of Stat1 and Stat2 proteins were found to be strongly inhibited in all replicon cell lines. Taken together our results suggest that the lack of phophoryated STAT may be due to the reduced expression of Jak-1 and Tyk2 in resistant replicons. Our data suggests that the defect in Jak-Stat signaling can contribute to the interferon resistant phenotypes.

While these studies are in progress, there are other laboratories also reported the development IFN-resistant replicon cell lines. Studies by Sumpter et al [41] suggest that a mutated replicon upon high passage develops resistance to interferon. This suppression was due to a reduced activation of IFN-stimulated gene expression and blockage at the viral IRES translation. Namba et al [42] developed an IFN-resistant replicon by prolonged treatment with low doses of IFN-α. These investigators have examined the genetic alteration associated with the interferon resistance. They found amino acid substitution in the NS4B and several amino acid substitutions in the NS5A regions suggesting that mutation in the viral sequence are involved in the IFN-resistance. Subsequent studies by the same group by Naka et al [43] reported that interferon resistance in the replicon cells caused by functional disruption of type I interferon receptor gene (IFNAR1 and IFNAR2c). Another study by Zhu et al [44] suggested that mutation in the viral sequence is not responsible for interferon resistance rather interferon resistance is due to a defect in the Stat 3 activation. In this report the authors did not notice any differences in the Stat1 and Stat2 phosphorylation. Our results suggest that a specific defect in the expression of components in the Jak-Stat pathways leads to defective Stat1 and Stat 2 phosphorylation. Because of these defects, replicon cells are unable to transmit signal to the nucleus and unable to induce antiviral gene expression by interferon. The underlying mechanisms of reduced expression of Tyk2 and Jak1 proteins in these resistant cell clones are under investigation. We propose that examining the intracellular interferon signaling pathways using IFN-sensitive and resistant hepatocytes from chronically infected humans may provide critical information regarding the mechanisms of interferon resistance in the chronic hepatitis C.

## Methods

### Replicon Cells

Human hepatoma cell line Huh-7 cells were obtained from the laboratory of James Wilson, Wistar Institute of Human Gene Therapy, Pensylvania, grown in Dulbecco's Modified Eagle's Medium (D-MEM), supplemented with 10% fetal bovine serum (FBS), non-essential amino acids and sodium pyruvate. Stable replicon cell lines (Con-15, Con-17, Con-24) were prepared in our laboratory as described earlier [38]. Stable HCV replicon cell lines 5–15 and 9–13, replicating HCV subgenomic RNA were obtained from the laboratory of Ralf Bartenschlager, Germany. Another HCV replicon cell line (KR) was obtained from George Liu, University of Kentucky. All replicons cell lines were cultured in presence of G-418 (1 mg/ml, Geniticine, Invitrogen Life Technologies, Carlsbad, California, USA).

### IFN Treatment

Three different replicon cell lines (9–13, 5–15 and KR) showing higher activation of interferon promoter and three different replicon cell lines (Con-15, Con-17 and Con-24) showing a low level activation of interferon promoter were cultured in 100-mm culture dishes. All the replicon cells were treated with human recombinant IFN-α2b (10–1000 IU/ml) (Intron-A, Schering Plough Co., New Jersey, USA) in growth medium supplemented with 1 mg/ml G-418 in order to select cell colonies that are truly resistant to interferon. Cultures were maintained for more than two months with a regular medium change at 3 days until apparent IFN-resistant cell colonies developed on the culture plate. After 4 weeks of culture, IFN-resistant cell clones were picked up and stable cell lines were generated.

### Replication assay

The ability of each of these replicon cell lines to resist the antiviral action of interferon was examined by measuring G-418 resistant cell colonies, sustained expression of viral protein and replication of HCV RNA in the presence of IFN-α2b. Both resistant and sensitive replicon cells were cultured in 100-mm tissue culture dishes using a growth medium containing 1 mg/ml G-418 with IFN-α2b (1000 IU/ml). The cells were maintained with a regular medium change at every third day for a month in the presence of interferon. The appearance of resistant cell colonies on the tissue culture dishes was recorded. These results were directly compared with interferon sensitive cell lines.

### Ribonuclease Protection assay

To examine whether HCV-RNA replication in the replicon cells was resistant to the antiviral action of interferon, cells were cultured in the presence of IFN-α2b (1000 IU/ml). Total RNA was isolated from the transfected cells after a week by the GITC method. HCV positive strand RNA was detected by a ribonuclease protection assay using an antisense riboprobe targeted to the highly conserved 5' UTR region. These results were directly compared with interferon sensitive cell lines. The plasmid pCR II-296 was linearized with *Xba I *and used to prepare an anti-sense RNA probe using the SP6 RNA polymerase. For RPA assays, approximately 1 × 10^6 ^cpm of the ^32^P-labeled anti-sense probe was added to 25 μg of RNA sample and then vacuum dried. Hybridization was performed in 10 μl of the hybridization buffer after denaturing for 3 minutes at 95°C and followed by overnight incubation at 45°C. RNase digestion was performed in 200 μl of RNase cocktail (1: 100) (Ambion Inc. Austin, Texas) in a buffer consisting of 10 mM Tris, pH 7.5, 5 mM EDTA and 0.3 M NaCl for 1 hour at 37°C. Reactions were stopped by the addition of 2.5 μl of 25% SDS and 10 μl of proteinase K (10 mg/ml) at 37°C for 15 minutes. Samples were extracted with phenol/chloroform and precipitated with ethanol. The pellet was air dried and resuspended in 15 μl of gel loading buffer. The samples were then boiled for 3 minutes and separated on an 8% acrylamide/8 M urea gel. The gel was dried and exposed to X-ray film (Kodak, X-OMAT-AR).

### Viral protein expression

The level of viral NS3 protein expression in the resistant cells was examined by an immunocytochemical method using a monoclonal antibody. Replicon cells were immobilized onto glass slides by cytospin method. Cells were washed with phosphate-buffered saline (PBS) pH 7.4 twice, air-dried and fixed with chilled acetone for five minutes. The cells were permeabilized by treatment with 0.05% saponin for 10 minutes at room temperature. Blocking was performed with 5% normal goat serum (Sigma Chemical Company, St. Louis, MO) diluted in minimum essential medium for 30 minutes at room temperature. Blocking for endogenous biotin-avidin was performed using a commercially available kit (Avidin/Biotin Blocking Kit, Vector Laboratories Inc., Burlingame, CA). Blocking for endogenous peroxidase was carried out with 0.9% H_2_O_2 _for 30 minutes at room temperature. The cells were incubated with monoclonal anti-NS3 antibody (1:100 dilution) overnight at 4°C. The slide was then washed three times and incubated with anti-mouse biotin conjugated antibody (1:1000) for one hour at room temperature. The slides were then washed and incubated for 30 minutes with Elite avidin-biotin peroxidase complex (VECTOR Labs, CA). The slides were reacted with diaminobenzidine for 10 minutes. Counterstaining was performed with hematoxylin for one minute. After dehydration, the slides were mounted with permount and observed by light microscopy.

### Cyclosporin A treatment

Replication of sub-genomic HCV RNA in each replicon cell line was eliminated after treatment with cyclosporin A (1 mg/ml). Replicon cells were seeded in 100-mm plates and treated with cyclosporine A (1 mg/ml) (Sigma Chemical Co. St. Louis, Mo., USA) for one week in growth medium without G-418. Presence or absence of HCV in these cells was examined by expression of NS3 and viral RNA by RPA. We selected cyclosporine A because this drug inhibits HCV replication without any effect on the ISRE promoter activity [37]. Interferon resistant phenotypes in these cured cells were examined by measuring their ability to activate interferon promoter and HCV IRES mediated translation of GFP by the addition of exogenous IFN-alpha2b.

### Luciferase assay for IFN-β promoter

Regulation of ISRE-driven transcription of firefly luciferase gene by IFN α was studied using IFN-sensitive and IFN-resistant cell lines. Cells were transfected with 1 μg of pISRE-luciferase plasmid (pISRE-Luc) (Fig. 1B) using the FuGENE 6 transfection reagent (Roche Diagnostic Corporation, Indianapolis, Ind., USA). IFN-α2b (1000 IU/ml) was added to the transfected cells to study its effect on ISRE-mediated transcription of luciferase gene. To measure luciferase activity, cells were lyzed in a reporter lysis buffer (Promega Corporation, Madison, Wisconsin, USA) according to the manufacturer's instructions. The level of expression in the replicons cell clones from the ISRE promoter was carefully examined after correcting for the amount of proteins in the lysates and the differences in efficiencies of transfection. Luciferase activity was measured by integrating the total light emission over 10 sec with a luminometer (Luman LB9507, EG&G Berthold, Berlin, Germany). The results of RLU among transfected cells were compared and values were expressed as fold induction compared with the mock-transfected Huh-7 cells. All experiments were done in triplicates as described previously [37].

### HCV IRES-GFP translation

Interferon action on HCV IRES mediated translation of green fluorescence protein was examined by using IFN-sensitive and IFN-resistant cell clones. HCV IRES-GFP expression in each cured Huh-7 cell line was performed using two-step transfection procedures. Briefly, cells were infected with 2 μl of the replication defective adenovirus carrying the gene for T7 RNA polymerase. After 2 hours, cells were transfected with 1 μg of pHCV-IRES-GFP plasmid (Fig. 1C) using FuGENE 6 transfection reagent (Roche Diagnostic Corporation, Indianapolis, Ind., USA). Immediately after, cells were incubated for 24 hours with or without addition of IFN α-2b (1000 IU/ml). Cells were counterstaining with DAPI (Calbiochem, San Diego, CA). Expression of GFP in the transfected cell was examined using a fluorescent microscope and composite picture was generated by Adobe Photoshop computer software.

### Western Blot Analysis

Cell lysates were prepared from replicon cells and examined for the expression of Jak-Stat signaling protein by Western blot analysis. Antibodies for Jak-1, Tyk2, Stat 1, Stat 2, Stat 3 proteins and phosphorylated Stat 1 and Stat 2 proteins were obtained from Cell Signaling Technology, Beverly, MA. Antibody to interferon receptor was obtained from R & D systems. Polyclonal antibody to interferon receptor was obtained from Santa Cruz Laboratory. Antibody against beta actin was obtained from Sigma Chemical Co, Saint Louis. Cured IFN-sensitive and resistant replicons were treated with recombinant human IFN-α (1000 IU/ml) for 30 minutes and Western blot analysis for individual protein was performed using a standard procedure of our laboratory [38].

### IFN receptor binding assay

To determine whether interferon resistance phenotypes in these resistant cells could have occurred due to lack of expression or deletion of functional receptors. Interferon binding to cell surface receptors was compared between sensitive and resistant cells. For this purpose, IFN α-2b (INTRON A, Schering Corporation) was labeled with ^125^I using Iodobeads following the manufacturer's instructions (Pierce, Rockford, IL. USA) as previously described [45,46]. Five micrograms of IFN-α were incubated with 10 μCi of NaI 125 (ICN Biochemicals) for 15 minutes. Free and protein-bound ^125^I were separated by elution through a prepacked Sepharose G-25 column (Pharmacia PD-10). Peak fractions of radioactivity were pooled and the specific activity was determined (radioactivity associated with per microgram of interferon). Binding experiments were performed using a standard procedure described previously [45]. Hundred microliter of cured Huh-7 cells (10^5 ^cells) were incubated with six different concentrations of ^125^I-IFN α in 1.5 ml conical tubes and incubated for 60 minutes at 37°C. After centrifugation to 12000 rpm × 5 minutes cell the pellet was washed with 500 μl of PBS, twice, and resuspended in 100 μl of PBS. The radioactivity was detected by one minute in a gamma counter (LKB Wallac-1282 Compugamma Universal Gamma Counter). Nonspecific binding (NSB) was measured in presence of 100-fold excess of unlabelled IFN-α2b for each dilution. The specific binding of interferon to Huh-7 cells at a different concentration was recorded. The amount of radioactivity specifically bound to the cell surface at each concentration of interferon was determined.

## Competing interests

The author(s) declare that they have no competing interests.

## References

[B1] Alter HJ, Seeff LB (2000). Recovery, persistence and sequelae in hepatitis C virus infection: a perspective on long-term outcome. Seminar Liver Disease.

[B2] Lauer G, Walker B (2001). Medical progress: hepatitis C virus infection. New Eng J Med.

[B3] Alter MJ (1997). Epidemiology of hepatitis C. Hepatology.

[B4] Liang TJ, Rehermann B, Seeff LB, Hoofnagle JH (2000). Pathogenesis, natural history, treatment, and prevention of hepatitis C. Ann Intern Med.

[B5] Hoofnagle JH (2004). Hepatocellular carcinoma: Summary and recommendation. Gastroenterology.

[B6] El-Serag HB (2004). Hepatocellular carcinoma: recent trends in the United States. Gastroenterology.

[B7] Davis GL (2000). Current therapy for chronic hepatitis C. Gastroenterology.

[B8] Brown RS (2005). Hepatitis C and liver transplantation. Nature.

[B9] Davis GL, Esteban-Mur R, Rustgi V, Hoefs J, Gordon SC, Trepo C, Shiffman ML, Zeuzem S, Craxi A, Ling MH, Albrecht J (1998). Interferon alfa-2b alone or in combination with ribavirin for the treatment of relapse of chronic hepatitis C. International Hepatitis Interventional Therapy Group. N Engl J Med.

[B10] Manns MP, McHutchison JG, Gordon SC, Rustgi VK, Shiffman M, Reindollar R, Goodman ZD, Koury K, Ling M, Albrecht JK (2001). Peginterferon alpfa-2b plus ribavirin compared with interferon alfa-2b plus ribavirin for initial treatment of chronic hepatitis C: a randomized trial. Lancet.

[B11] Feld JJ, Hoofnagle JH (2005). Mechanism of action of interferon and ribavirin treatment of hepatitis C. Nature.

[B12] Strader DB, Wright T, Thomas DL, Seeff LB, American Association for the Study of Liver Diseases (2004). Diagnosis, management, and treatment of hepatitis C. Hepatology.

[B13] Fried MW, Shiffman ML, Reddy KR, Smith C, Marinos G, Goncales FL, Haussinger D, Diago M, Carosi G, Dhumeaux D, Craxi A, Lin A, Hoffman J, Yu J (2002). Peginterferon alfa-2a plus ribavirin for chronic hepatitis C virus infection. New Eng J Med.

[B14] Simmonds P (2004). Genetic diversity and evolution of hepatitis C virus–15 years on. J Gen Virol.

[B15] Bukh J, Miller RH, Purcell RH (1995). Genetic heterogeneity of hepatitis C virus: quasispecies and genotypes. Semin Liver Dis.

[B16] Reed KE, Rice CM (2000). Overview of hepatitis C virus genome structure, polyprotein processing and protein properties. Curr Top Microbiol Immunol.

[B17] Pawlotsky JM (2003). The nature of interferon-alpha resistance in hepatitis C virus infection. Current Opinion on Infectious Disease.

[B18] Pawlotsky JM (2003). Mechanisms of antiviral treatment efficacy and failure in chronic hepatitis C. Antiviral Research.

[B19] Enomoto N, Sakuma I, Asahina Y, Kurosaki M, Murakami T, Yamamoto C, Izumi N, Marumo F, Sato C (1995). Comparison of full-length sequences of interferon-sensitive and resistant hepatitis C virus 1b. Journal of Clinical Investigation.

[B20] Enomoto N, Sakuma I, Asahina Y, Kurosaki M, Murakami T, Yamamoto C, Ogura Y, Izumi N, Marumo F, Sato C (1996). Mutation in the nonstructural protein 5A gene and response to interferon in patients with chronic hepatitis C virus 1b infection. New Eng J Med.

[B21] Paterson M, Laxton CD, Thomas HC, Ackrill AM, Foster GR (1999). Hepatitis C virus NS5A protein inhibits interferon antiviral activity but the effects do not correlate with clinical response. Gastroenterology.

[B22] Hoffmann WP, Zeuzem S, Sarrazin C (2005). Hepatitis C virus-related resistance mechanisms to interferon alpha-based antiviral therapy. Journal of Clinical Virology.

[B23] Schinkel J, Spoon WJ, Kroes AC (2004). Meta-analysis of mutations in the NS5A gene and hepatitis C virus resistance to interferon therapy: uniting discordant conclusions. Antiviral Therapy.

[B24] Nousbaum J, Polyak SJ, Ray SC, Sullivan DG, Larson AM, Carithers RL, Gretch DR (2000). Prospective characterization of full-length hepatitis C virus NS5A quasispecies during induction and combination antiviral therapy. Journal of Virology.

[B25] Gale MJ, Korth MJ, Tang NM, Tan SL, Hopkins DA, Dever TE, Polyak SJ, Gretch DR, Katze MG (2000). Evidence that hepatitis C virus resistance to interferon is mediated through repression of the PKR protein kinase by the nonstructural 5A protein. Virology.

[B26] Gale M, Blakely CM, Kwieciszewski B, Tan SL, Dossett M, Tang NM, Korth MJ, Polyak SJ, Gretch DR, Katze MG (1997). Control of PKR protein kinase by hepatitis C virus non-structural 5A protein: Molecular mechanisms of kinase regulation. Molecular and Cellular Biology.

[B27] Taylor DR, Shi ST, Romano PR, Barber GN, Lai MM (1999). Inhibition of the interferon-inducible protein kinase R by HCV E2 protein. Science.

[B28] Blindenbacher A, Duong FH, Hunziker L, Stutvoet ST, Wang X, Terracciano L, Moradpour D, Blum HE, Alonzi T, Tripodi M, La Monica N, Heim MH (2003). Expression of hepatitis C virus proteins inhibits interferon alpha signaling in the liver of transgenic mice. Gastroenterology.

[B29] François C, Duverlie G, Rebouillat D, Khorsi H, Castelain S, Blum HE, Gatignol A, Wychowski C, Moradpour D, Meurs EF (2003). Expression of hepatitis C virus proteins interferes with the antiviral action of interferon independently of PKR-mediated control of protein synthesis. Journal of Virology.

[B30] Keskinen P, Melen K, Julkunen I (2003). Expression of HCV structural proteins impairs IFN-mediated antiviral response. Virology.

[B31] Lin W, Choe WH, Hiasa Y, Kamegaya Y, Blackard JT, Schmidt EV, Chung RT (2005). Hepatitis C virus expression suppresses interferon signaling by degrading STAT1. Gastroenterology.

[B32] Gale M, Foy EM (2005). Evasion of intracellular host defence by hepatitis C virus. Nature.

[B33] Kawai T, Akira S (2006). Innate Immune recognition of viral infection. Nature Immunol.

[B34] Uze G, Lutfalla G, Gresser I (1990). Genetic transfer of a functional human interferon alpha-receptor into mouse cells: cloning and expression of its cDNA. Cell.

[B35] Darnell JE (1998). Studies of interferon-induced transcriptional activation uncover the Jak-STAT pathway. J of Interf and Cytok Res.

[B36] Goodbourn S, Didcock L, Randall RE (2000). Interferons: cell signaling, immune modulation, antiviral responses and virus countermeasures. J of Gen Virol.

[B37] Pai M, Prabhu R, Panebra A, Nangle S, Haque S, Bastian F, Garry R, Agrawal K, Goodbourn S, Dash S (2005). Activation of interferon stimulated response element (ISRE) in Huh-7 cells replicating HCV subgenomic RNA. Intervirology.

[B38] Dash S, Prabhu R, Hazari S, Bastian F, Garry R, Zou W, Haque S, Joshi V, Regenstein FG, Thung SN (2005). Interferons alpha, beta, gamma each inhibits hepatitis C virus replication at the level internal ribosome entry site mediated translation. Liver International.

[B39] Reddy KR, Hoofnagle JH, Tong MJ (1999). Racial differences in responses to therapy with interferon in chronic hepatitis c. Consensus Interferon Study Group. Hepatology.

[B40] Gao B, Hong F, Radaeva S (2004). Host factors and failure of interferon alpha treatment in hepatitis C virus. Hepatology.

[B41] Sumpter R, Wang C, Foy E, Loo YM, Gale M (2004). Viral evolution and interferon resistance of hepatitis C virus RNA replication in a cell culture model. J of Virol.

[B42] Namba K, Naka K, Dansako H, Nozaki A, Ikeda M, Shiratori Y, Shimotohno K, Kato N (2004). Establishment of hepatitis C virus replicon cell lines possessing interferon-resistant phenotype. Biochem and Biophys Res Comm.

[B43] Naka K, Takemoto K, Abe K, Dansako H, Ikeda M, Shimotohno K, Kato N (2005). Interferon resistance of hepatitis C virus replicon-harbouring cells is caused by functional disruption of type1 interferon receptors. J of Gen Virol.

[B44] Zhu H, Nelson D, Crawford JM, Liu C (2005). Defective Jak-Stat activation in hepatoma cells is associated with hepatitis C viral IFN-alpha resistance. J of Interf and Cytok Res.

[B45] Kimball P, Verbeke S, Shiffman M (2003). Comparison of ^125^I-interferon-alpha binding to peripheral blood cells from African-Americans and Caucasians with hepatitis C. J Viral Hepat.

[B46] Branca A, Faltynek C, D Alessandro, Baglioni C (1982). Interaction of interferon with cellular receptors: internalizationand degradation of cell-bound interferon. J Biol Chem.

